This article has been retracted.

# Network Pharmacology‐Based Study on the Active Component and Mechanism of the Anti-Gastric-Cancer Effect of *Herba Sarcandrae*

**DOI:** 10.1155/2021/3001131

**Published:** 2021-11-19

**Authors:** Li Han, Ying Han

**Affiliations:** ^1^The Third Hospital of Hebei Medical University, Pharmacy Department, Shijiazhuang, China; ^2^The Third Hospital of Hebei Medical University, Department of Chinese Medicine, Shijiazhuang, China

## Abstract

**Background:**

*Herba Sarcandrae* is used in the clinical practice of traditional Chinese medicine to deal with gastric cancer. However, there are few studies on its precise mechanism.

**Method:**

In this study, a network pharmacological approach was utilized to construct a molecular/target/pathway molecular regulatory network for the anti-gastric-cancer effect of *Herba Sarcandrae*. The active components of *Herba Sarcandrae* and their potential mechanisms were explored. Chemical components of the *Herba Sarcandrae* were identified through a database, and they were evaluated and screened based on oral bioavailability and drug similarity.

**Results:**

Genes related to gastric cancer were found in the Gene Expression Omnibus (GEO) database, and gene targets related to anti-gastric-cancer were chosen by comparison. Using annotation, visualization, and a comprehensive discovery database, the function and related pathways of target genes were analyzed and screened. Cytoscape software was utilized to construct a component/target/pathway network for the antitumor effect of *Herba Sarcandrae*. Finally, 6 drug ingredients and 29 target genes related to gastric cancer were detected. IL-17 signaling pathway, NF-kappa B signaling pathway, and other signaling pathways were significantly enriched. Many signaling pathways that directly act on tumors and indirect pathways inhibit the development of gastric cancer.

**Conclusion:**

This study provides a scientific basis for further elucidating the mechanism of the anti-gastric-cancer effect of *Herba Sarcandrae*.

## 1. Introduction

Gastric cancer is among the most common malignant tumors in the world, and its morbidity and mortality rank fourth and second, respectively, in cases where cancer has been clearly diagnosed [1]. Because gastric cancer is a highly aggressive tumor, there are many specific symptoms and signs at an early stage, making it difficult for patients to pay attention to and be diagnosed by doctors in a timely manner, and it is late when it is discovered. Although the current preliminary screening, surgical resection, and chemotherapy have significantly improved the clinical efficacy of gastric cancer, the 5-year survival rate of gastric cancer patients is less than 30% [2]. In addition, the high cost of treatment has placed a heavy financial burden on patients with gastric cancer [3]. Therefore, there is an urgent need to develop new anti-gastric-cancer drugs that have useful anticancer activity and low toxic and side effects.

In recent years, the active ingredients of native plants have attracted more and more attention in cancer prevention and treatment due to their low toxicity, broad spectrum, and high efficiency [4]. *Acorus veterinarians* can inhibit human glioma cell proliferation through p53 [5]. In terms of inducing apoptosis, the effective ingredient of origin can induce endogenous apoptosis of gastric cancer cells through the peripatetic factors Apaf-1, caspase-3, and Cyto C [6]. Ophiophagus B can induce autophagy and mitotic death of non-small cell lung cancer A549 cells [7]. Danshen injections can directly inhibit mutant JAK2 and its protein phosphorylation, thereby inhibiting the proliferation of erythroid leukemia cells with JAK2 mutation [8]. Thus, traditional Chinese medicine has an important additional option for the development of innovative cancer treatments.

*Herbal Sarcandrae* is the whole plant of *Sarcandra glabra* (Thunb.) Nakai, a plant of the family Nasturtium, and has become one of the key Chinese medicines to be discovered in China. Chemical components of *Herba Sarcandrae* are mainly flavonoids, coumarins, organic acids, polysaccharides, volatile oils, and sesquiterpenes [9, 10]. With a good antitumor effect of *Herba Sarcandrae* clinically, more and more *Herba Sarcandrae* preparations are also widely used in the treatment of tumors. For example, *in vitro* experiments have found that *Herba Sarcandrae* on human liver cancer cells HepG2, [11] human prostate cancer cells PC-3, human breast cancer cells MCF-7, [12] human lung cancer A-549, colon cancer HCT-29, and gastric cancer BGC-82 has a strong cytotoxic effect and is dose-dependent [13]. *In vivo* experiments found that human gastric cancer SGC-7901 tumor cells inoculated into nude mice formed apoptosis bodies after continuous administration of Zhongjiefeng injection for 14 days. The doses of the drug on human gastric cancer SGC-7901 xenografts in nude mice were 42.8% and 39.9%, respectively [14]. *Herba Sarcandrae* has a variety of anticancer components and has definite antitumor effects. However, the mechanism and molecular target of *Herba Sarcandrae* in treating gastric cancer are unclear, which is the principal factor limiting its widespread application.

Traditional Chinese medicine is unique sanitation, economic, cultural, and biological resource in China. For thousands of years, it has served the Chinese nation's reproduction and prosperity and made significant contributions to the health of China. Single Chinese medicine therapy is a method with single traditional Chinese medicine as a prescription to treat various diseases and has a major impact. In the *Compendium* of *Materia Medica*, there are more than 2000 important single Chinese medicine prescriptions, many of which are still in clinical application. However, there are still numerous ingredients in definite Chinese medicine, and they also face huge challenges in clarifying the interactions between the ingredients, their action mechanisms, and molecular mechanisms. Network pharmacology is a novel method for predicting the mechanism of drug treatment of disease at the overall level by searching the network database, constructing the “drug-target-disease” network relationship, and performing network topology analysis. It integrates bioinformatics, multidirectional pharmacology, and other multidisciplinary technologies and content, starting from multitarget research strategies, achieving comprehensive network analysis of drug effects. Because of its holistic and systemic characteristics, network pharmacology has been broadly used for the prediction of potential active ingredients and targets of traditional Chinese medicine and the study of its mechanism of action [15]. Network pharmacology's research in lone Chinese medicine is mainly reflected in forecasting its possible targets and pathways through the known efficacy of Chinese medicine and in the process of verification, clarifying its action pathway. Li explored the mechanism of *Radix Puerariae* on coronary heart disease using network pharmacology. Through the network pharmacology method, it was discovered that *Radix Puerariae* exerts its therapeutic effect on coronary heart disease through multiple targets and multiple pathways. The nitric oxide pathway, AGE/RAGE pathway, and the anachronic acid pathway may be the major pathways for *Radix Puerariae* treatment of coronary heart disease [16]. Zhao studied the mechanism of *Chuanxiong Rhizoma* on coronary heart disease based on network pharmacology. It was noteworthy that *Chuanxiong Rhizoma* may treat coronary heart disease mainly by antioxidation, anti-inflammatory, anticoagulation, promoting angiogenesis, dilating blood vessels, and regulating blood pressure [17]. Li applied the network pharmacological method to predict the target and related signal pathways of *Spica Prunellae* against breast cancer and to explore its mechanism of anti-breast-cancer effect. *Spica Prunella* can exert anti-breast-cancer effects through targets such as estrogen receptors, cell-specific cycling, and epidermal growth factor receptors, as well as related pathways [18]. The previously mentioned studies showed that network pharmacology has gradually started to penetrate into various aspects of research in the field of traditional Chinese medicine, exploring new aspects of traditional Chinese medicine and systematically explaining the ingredient-target relationship and pharmacological mechanism of single traditional Chinese medicine or compound traditional Chinese medicine. Collecting traditional Chinese medicine ingredients and predicting the target of the action, clarifying the action mechanism of single Chinese medicine, and discovering the latest indications of traditional Chinese medicine have critical application value.

In this study, a network pharmacological approach was to be used to explore the mechanism of action and molecular targets of *Herba Sarcandrae* for gastric cancer. Our protocol is shown in Figure 1. The active compounds of *Herba Sarcandrae* and their targets were first identified using the TCMSP database. Gastric-cancer-related targets were then obtained by analyzing differentially expressed genes between patients with gastric cancer and healthy individuals. Through the analysis of gene ontology (GO) and Kyoto Encyclopedia of Genes and Genomes (KEGG) pathways, the probable mechanism of the treatment of gastric cancer by *Herba Sarcandrae* was analyzed, which had a theoretical reference for subsequent pharmacological related research. It will be important to investigate the mechanisms of traditional Chinese medicine, drug targets, and discovery and provide a reference for future clinical practices.

## 2. Materials and Methods

### 2.1. Active Ingredient Screening

We identified chemical constituents of *Herba Sarcandrae* from the Traditional Chinese Medicine Systems Pharmacology Database, and Analysis Platform (TCMSP, https://lsp.nwu.edu.cn/tcmsp.php) [19]. This database is used to obtain the composition information, including composition number, molecular name, molecular weight, fat-water partition coefficient, number of hydrogen bond donor acceptors, oral bioavailability (OB), intestinal epithelium permeability, blood-brain barrier (BBB), drug similarity (DL), and drug half-life (HL). We chose to have oral bioavailability (OB) ≥30% and drug similarity (DL) ≥0.18 [20].

### 2.2. Identify Potential Targets

These 10 candidate compounds were imported into the DrugBank database (https://www.drugbank.ca/) to identify the corresponding targets of *Herba Sarcandrae*. After removing 1 compound that was not related to any target, 9 compounds were finally selected [21].

### 2.3. Targets Related to Gastric Cancer

Differentially expressed genes in gastric cancer patients were obtained from the GEO database (https://www.ncbi.nlm.nih.gov/geo/), series: GSE118916, number of samples: GSM3351235-3351249 are normal samples, GSM3351220-3351234 are gastric cancer samples. Genes with adjusted *P* values < 0.05 and |log 2 (FC)| >1 were considered to be significantly differentially expressed and related to gastric cancer.

### 2.4. Network Construction

Search Tool for the Retrieval of Interacting Genes database (version 10.0, https://string-db.org) was used to predict potential interactions between target candidates at the protein level. A combined score of >0.4 (medium confidence score) was considered significant. Additionally, Cytoscape software (version 3.7.2, https://www.cytoscape.org/) was utilized for constructing the PPI network. Degree ≥20 was set as the cutoff criterion. The Molecular Complex Detection (MCODE) app was used to analyze PPI network modules, [22] and MCODE scores >3 and the number of nodes >5 were set as cutoff criteria with the default parameters (degree cutoff ≥2, node score cutoff ≥2, K-score ≥2, and Max depth = 100). Finally, CytoHubba, a Cytoscape plugin, was utilized to explore PPI network hub genes; it provides a user-friendly interface to explore important nodes in biological networks and computes, using eleven methods, of which MCC has a better performance in the PPI network [23].

### 2.5. Gene Ontology (GO) and KEGG Pathway Enrichment Analysis

The Kyoto Encyclopedia of Genes and Genomes (KEGG) approach is a knowledge base for the systematic analysis of gene function [24]. The Database for Annotation, Visualization and Integrated Discovery (DAVID) provides researchers with a comprehensive and effective set of concise annotation tools to help them understand the biological significance behind many genes [25]. The DAVID was used for GO and KEGG pathway enrichment analysis for DEG. FDR <0.05 was fixed as the cutoff standard for two analyses.

### 2.6. Prognostic Analysis of Key Genes

The Cancer Genome Atlas (TCGA) database is a collaborative project between the National Human Genome Research Institute (NHGRI) and the National Cancer Institute (NCI). By sequencing, TCGA performed a genomic analysis of 33 tumors. This study uses gastric cancer groupings in the TCGA database to discuss the prognosis of core genes and draw Kaplan-Meier survival curves to examine the relationship between the expression of key genes and the prognosis of gastric cancer.

## 3. Results

### 3.1. Screening of Active Components

Results of oral bioavailability and drug similarity screening showed 10 compounds as candidate compounds (Table 1). 1143 genes associated with gastric cancer were identified from the GEO database. As shown in Figure 2, a volcano plot was created in order to provide evidence of the distribution of differentially expressed genes, of which 511 genes were upregulated and 632 genes were downregulated. The ingredient targets network of *Herba Sarcandrae* is constructed according to the screened ingredients and their targets, as shown in Figure 3. The network contains 35 points (6 ingredients- and 29 ingredients-targets in *Herba Sarcandrae*) and 40 edges, indicating compound-target interactions.

### 3.2. Identifying Candidates for *Herba Sarcandrae* for Gastric Cancer

Overlapping targets indicated a distinct set of interactions and networks. The PPIs for combining scores greater than 0.4 were selected for constructing PPI networks. The entire PPI network was analyzed using MCODE, following which one module was chosen (Figure 4). The first 10 genes in the MCC method were selected by the CytoHubba plugin and sequentially ordered as follows: IL-6, MMP9, HMOX1, PTGS2, CCL2, CXCL10, SPP1, ICAM1, VCAM1, and SERPINE1 (Figure 5).

### 3.3. GO and KEGG Enrichment Analysis

DAVID was utilized to perform GO and KEGG pathway enrichment analysis on 29 drug targets of identifying gastric cancer. Based on biological processes, cellular components and molecular functions were analyzed for candidate target GO. As shown in Figure 6, 590 GO terms were significantly enriched in gastric cancer (FDR <0.05), 475 in biological processes, 18 in cellular components, and 22 in molecular functions. GO terms that are highly enriched in biological processes, cellular components, and molecular functions include response to tumor necrosis factor, regulation of epithelial cell apoptosis process, mononuclear cell migration, and myeloid leukocyte migration. KEGG enrichment analysis of these drugs-targets genes identified 33 functional pathways exhibiting significant enrichment (Figure 7), including TNF signaling pathway, IL-17 signaling pathway, and NF-kappa B signaling pathway.

### 3.4. Genetic Pathway Network Analysis

A gene pathway network was constructed based on significantly rich pathways and the genes that regulate these pathways, as shown in Figure 8. Topological analysis of 20 pathways and 23 genes was carried out using BC in gastric cancer. The round rectangle represented target genes, and the V-shapes represented pathways in the network. The network diagram suggested that IL-6 had the maximum BC and was at the heart target gene. Further several genes also had larger BC, such as PRKCB, ICAM1, VCAM1, MYC, and CCL2. They might be the main target genes for *Herba Sarcandrae* against gastric cancer.

### 3.5. Analysis of Gene Prognosis of Drug-Targets

The TCGA database contains expression and clinical data on 33 types of tumors. Using TCGA database for prognosis analysis to investigate the effect of core genes on gastric cancer prognosis, survival analysis showed that the total survival of patients with high gene expression of IL-6, COL1A1, PTGS2, SELE, VCAM1, and SERPINE1 was lower than that of low expression patients, the difference was statistically significant (log-rank *P* < 0.05), and the difference in the results of other genes was not statistically significant (Figure 9).

## 4. Discussion

At present, tumors have formed part of the most serious diseases that endanger human health. It was estimated that, by 2020, there would be more than 20 million deaths caused by tumors worldwide. The incidence of tumors in China is also increasing year by year [26]. Traditional Chinese medicine has played an important role in the prevention and treatment of tumors, and its role and mechanism in enhancing the body's immune function, reversing multidrug resistance of tumor cells, inhibiting tumor cell division and proliferation, and accelerating tumor cell apoptosis have been gradually revealed. The effective application in antitumor laid the groundwork [27]. However, the composition of traditional Chinese medicine is complicated, and its active ingredients are unclear in pharmacology and clinical practice. Specific target genes or proteins for drug action have not been fully identified. In recent years, with the rapid development of high-throughput technology and bioinformatics, network pharmacology has got a solution to the problem of multicomponent/multitarget/complex disease of traditional Chinese medicine [28]. Research in network pharmacology in disease treatment has attracted global attention. Based on modern computer simulation technologies, it provides an effective method for component screening and prediction of drug targets.

In this study, we used network pharmacology methods to further explore the mechanisms of *Herba Sarcandrae* on gastric cancer. A total of 36 ingredients were found in the TCMSP database. We selected 10 major ingredients through OB and DL screening, including beta-sitosterol, sitosterol, anhydroicaritin, engeletin, Istanbulin-A, ZINC00391893, Chloranthalactone-A, (2R)-3-(3,4-dihydroxy phenyl)-2-[(Z)-3-(3,4-dihydroxy phenyl)acryloyl]oxy-propionic acid, and quercetin. Comparing the differences between gastric cancer genes and drug targets, we found 6 anti-gastric-cancer ingredients, beta-sitosterol, anhydroicaritin, engeletin, ZINC00391893, (2R)-3-(3,4-dihydroxy phenyl)-2-[(Z)-3-(3,4-dihydroxy phenyl)acryloyl]oxy-propionic acid, and quercetin, acquiring 29 key targets (Figure 2).

Moreover, we also use PPI to explore data mining and network analysis. We found 10 core targets (Figure 4). The GO enrichment analysis found targets involving the nucleus, cytoplasm, and other cellular compartments. At the molecular level, targets are associated with protein binding, energy metabolism, protein phosphorylation, and other molecular activities and are related to apoptosis, cell proliferation, and cell migration. Many gastric cancer studies have shown that the development of gastric cancer is a complex, multistep, and multifactor process, with a variety of potential risk factors, mainly genetic variation and environmental factors [29]. Environmental factors include *Helicobacter pylori* (HP) infection, eating habits, smoking, and drinking [30]. It has been reported that the expressions of antiapoptotic BCL2 and prostaglandin-endoperoxide synthase 2 (PTGS2) genes are abundant in gastric cancer and related to poor patient survival and are closely related to cisplatin resistance. Further research shows that PTGS2 participates in the development of cisplatin resistance by mediating the inhibitory effect of cisplatin on BCL2 expression [31]. In gastric cancer resistance studies, it was found that the combination of 6-ginger oil and cisplatin inhibited cell viability and enhanced cell cycle arrest in the G1 phase compared with cisplatin alone. Combination therapy inhibited cell migration and invasion, reduced cyclin D1, cyclin A2, matrix metalloproteinase-9, p-PI3K, AKT, and p-AKT protein expressions, and increased p21 and p27 mRNA levels. The development of gastric cancer is a dynamic process that interacts with the tumor microenvironment. Survival and migration of gastric cancer are closely related to the microenvironment [32–34]. Collagen is the key component of the extracellular mesenchyme of gastric cancer cells, and it is also the core component of the interstitial microenvironment. Collagen can provide growth, attachment, and a scaffold for tumor cells and induce migration of tumor cells [35, 36]. Evidence suggests that collagen synthesis increases during the development of gastric cancer [37]. In this study, we found that the expressions of the aforementioned collagen-related genes grew up in differential genes in gastric cancer. COL1A1 and COL3A1 may be the key genes implicated in the development of gastric cancer. Through drug-target interaction network analysis of the different genes, we found that the previously mentioned COL genes (including COL1A1) can be used as therapeutic targets for *Herba Sarcandrae*, indicating that *Herba Sarcandrae* can inhibit the expressions of these genes and affect the survival of gastric cancer and migration. Therefore, *Herba Sarcandrae* may play a regulatory role in the pathogenesis of gastric cancer and may affect some cellular components and molecular functions in the treatment of gastric cancer, including nucleus, cytoplasm, protein binding, enzyme binding, and DNA binding.

KEGG signaling pathway enrichment was found, and a total of 28 KEGG pathways, including IL-17 signaling pathway and NF-kappa B signaling pathway, were significantly enriched. The interleukin 17 (IL-17) family is a subset of cytokines composed of IL-17A-F and plays a key role in both acute and chronic inflammatory responses. The IL-17 family signals through its corresponding receptors and activates downstream pathways, including NF-*κ*B, MAPK, and C/EBP, to induce the expressions of antibacterial peptides, cytokines, and chemokines. In addition, IL-17 is also a CD4^+^ T cell-derived angiogenesis mediator, which plays a major role in stimulating angiogenesis by regulating the production of multiple proangiogenic factors (including vascular endothelial growth factor). IL-17A induces VEGF upregulation and neovascularization through STAT3-mediated signaling pathways. The expression level of VEGF is related to tumor progression and metastasis in gastric cancer tissues. Therefore, the effect of swelling and rheumatism in the treatment of gastric cancer may be through the pathway to block the expression of VEGF, which affects the progression and metastasis of gastric cancer [38]. Nuclear factor-*κ*B (NF-kappa B) is the common name of a family of transcription factors that act as dimmers and regulate genes involved in immunity, inflammation, and cell survival. It has been found that abnormal activation of the NF-*κ*B signaling pathway plays an essential role in the occurrence and metastasis of gastric cancer. *Herba Sarcandrae* may affect the occurrence and metastasis of gastric cancer by inhibiting the aberrant activation of the NF-*κ*B signaling pathway [39]. Regulation of these considerably enriched gastric cancer-related pathways may be one of the mechanisms for the treatment of gastric cancer by *Herba Sarcandrae*. A network of gene pathways needed to be based on studying the core target genes for the treatment of gastrointestinal tumors. Studies have demonstrated that migration and invasion are the leading causes of death in patients with gastric cancer. There is growing evidence that IL-6 can stimulate cancer cell invasion and is made in association with cancer development [40]. IL-6 can mediate the JAK-STAT3-VEGF-C signaling pathway to promote gastric cancer growth, invasion, and lymphangiogenesis [41]. In addition, the tumor microenvironment (TME) plays a major role in the pathogenesis of numerous cancers. IL-6 induces M2 macrophage differentiation (IL-10^high^TGF-*β*^high^IL-12p35^low^) by activating STAT3 phosphorylation, and IL-6 induces M2 macrophages to play a tumor-promoting role by promoting gastric cancer cell proliferation and tumor formation [42]. Cancer-associated fibroblasts (CAF) are another important part of the tumor microenvironment. They promote tumorigenesis by secreting growth factors, modifying the extracellular matrix, supporting angiogenesis, and suppressing antitumor immune responses. It has been established that IL-6 can protect gastric cancer cells through paracrine signaling and mediate the crosstalk between tumor cells and CAF by promoting fibroblast activation [43]. Therefore, IL-6 and its related signaling pathways may be promising targets for the treatment of gastric cancer growth and lymphangiogenesis. By comparison to normal tissues, SERCINE1 was markedly upregulated in gastric cancer tissues. Elevated expression of SERPINE1 results in shorter overall survival and can be employed as an independent prognostic factor in gastric cancer patients. In addition, the downregulation of SERPINE1 showed an inhibitory effect on the phenotype of gastric cancer cells and dramatically inhibited the Epithelial-Mesenchymal Transition (EMT) process. The overexpression of SERPINE1 gave the opposite result. These data suggest that SERPINE1 promotes the proliferation, invasion, and migration of gastric adenocarcinoma cells, suggesting that SERPINE1 can be seen as a novel biomarker for gastric adenocarcinoma treatment [44]. Therefore, *Herba Sarcandrae* can regulate different target genes and signal pathways to inhibit the proliferation and induce apoptosis in gastric cancer cells.

In summary, this study was conducted as a preliminary exploration of superior ingredients, superior targets, and effective pathways of *Herba Sarcandrae* with the help of network pharmacology. That is, it has further established that *Herba Sarcandrae* provides pharmacological effect against gastric cancer. With the help of network pharmacology, superior monomer components in *Herba Sarcandrae* can be further excavated, which may become the basis for the development of novel drugs, but this still has to be experimented with. It illustrates the antigastric cancer pharmacological mechanism of *Herba Sarcandrae*.

## Figures and Tables

**Figure 1:** Flowchart of experimental designs.

**Figure 2:** Volcano plot of differentially expressed genes in gastric cancer. The abscissa is the fold changes in gene expression and the ordinate represents the statistical significance of the variations in gene expression. The red dots represent significantly upregulated expressed genes. The green dots represent markedly downregulated expressed genes.

**Figure 3:** Ingredient-target network of *Herba Sarcandrae*. The pink ellipse represents targets; the green diamond represents the ingredients from *Herba Sarcandrae.*

**Figure 4:** PPI network analysis of target proteins. (a) shows the target protein PPI network of *Herba Sarcandrae* ingredients; (b) shows the MCODE analysis after the construction of *Herba Sarcandrae* target protein PPI.

**Figure 5:** The network of the first 10 genes. The first 10 genes of the MMC method were chosen using CytoHubba plugin. The more forward ranking is represented by a redder color.

**Figure 6:** Gene ontology terms of candidate targets of *Herba Sarcandrae* against gastric cancer. The top 20 GO functional categories with FDR <0.05 were selected.

**Figure 7:** KEGG pathway enrichment of candidate targets of *Herba Sarcandrae* against gastric cancer. Pathways that had significant changes of FDR <0.05 were identified. The size of the spot represents a number of genes and color represents FDR value.

**Figure 8:** Gene pathway network of *Herba Sarcandrae* against gastric cancer. The topological analysis of 20 pathways and 23 genes was carried out with betweenness centrality. The blue round rectangle represents target genes and the pink V-shapes represent pathways. Big size represents the larger betweenness centrality.

**Figure 9:** Prognostic curves of six hub genes. The prognostic significance of the hub genes in patients with gastric cancer, according to the Kaplan-Meier plotter database. (a) IL-6; (b) COL1A1; (c) PTGS2; (d) SELE; (e) VCAM1; (f) SERPINE1. The red lines represent patients with high gene expression, and blue lines represent patients with a low gene expression.

**Table 1:** Chemical information for the constituents of *Herba Sarcandrae*.

MOL ID	Ingredients	Structure	Molecular weight	OB (%)	DL
000358	Beta-sitosterol		414.79	36.91	0.75
000359	Sitosterol		414.79	36.91	0.75
004373	Anhydroicaritin		368.41	45.41	0.44
004568	Engeletin		434.43	36.27	0.7
007132	(2R)-3-(3,4-Dihydroxyphenyl)-2-[(Z)-3-(3,4-dihydroxyphenyl)acryloyl]oxy-propionic acid		360.34	109.38	0.35
007742	Istanbulin-A		264.35	80.1	0.2
007743	ZINC00391893		270.3	41.92	0.2
007744	Chloranthalactone-A		228.31	41.72	0.18
007747	Chloranoside-A		262.33	84.11	0.23
000098	Quercetin		302.25	46.43	0.28

## Data Availability

The data used to support this study are available from the corresponding author upon request.

## Abbreviations

TCMSP: Traditional Chinese Medicine Systems Pharmacology Database, and Analysis Platform
GEO: Gene Expression Omnibus
EMT: Epithelial-Mesenchymal Transition
MCODE: Molecular Complex Detection.
